This article has been retracted.

# Falling-Point Recognition and Scoring Algorithm in Table Tennis Using Dual-Channel Target Motion Detection

**DOI:** 10.1155/2021/5529981

**Published:** 2021-04-19

**Authors:** Bo Yang, Zijian Chang, Ying Chen

**Affiliations:** ^1^Northeastern University, Shenyang 110819, Liaoning, China; ^2^School of Physical Education, Northwest Minzu University, Lanzhou 730030, Gansu, China; ^3^Department of Basic Course, Wuhan Donghu University, Wuhan 430212, Hubei, China

## Abstract

In table tennis, the ball has numerous characteristics of high speed, small size, and changeable trajectory. Due to these characteristics, the human eye often cannot accurately judge the ball's movement and position, leading to the problem of precise detection of the ball's falling point and movement tracking. In sports, the use of machine learning for locating and detecting the ball and the use of deep learning for reconstructing and displaying the ball's trajectories are considered futuristic technologies. Therefore, this paper proposes a novel algorithm for identifying and scoring points in table tennis based on dual-channel target motion detection. The proposed algorithm consists of multiple input channels to jointly learn different features of table tennis images. The original image is used as the input of the first channel, and then the Sobel operator is used to extract the first-order derivative feature of the original image, which is used as the input of the second channel. The table tennis feature information from the two channels is then fused and sent to the 3D neural network module. The fully connected layer is used to identify the table tennis ball's drop point, compare it with a standard drop point, calculate the error distance, and give a score. We also constructed a data set and conducted experiments. The experimental results show that the method in this paper is effective in sports.

## 1. Introduction

In all kinds of ball sports, the ball has fast speed, small size, and a changeable trajectory. The human eye often cannot accurately judge the movement posture of the ball [1], and often there are problems that the ball's falling point cannot be accurately recognized and the movement track cannot be retained. The use of machine learning techniques to identify and locate the ball and computer vision [4–9] and deep learning techniques [10–14] to reconstruct and display the ball's trajectory is a futuristic application. It results in instant playback systems in table tennis matches due to merging technology and sports. In recent years, major sports events have introduced such auxiliary referee systems [2], which help humans overcome the visual limit, thereby ensuring the game's fairness. They also provide audiences with more exciting game broadcasts [3], thereby improving the entertainment of the game.

In the process of training, table tennis players can often play superfast ball speeds, changeable touch-offs, out-of-bounds, controversial balls, and so forth, but the impact of table tennis is fleeting. Even professional coaches often do. It is impossible to identify the true situation of the impact point accurately. Moreover, athletes have to perform a lot of training every day. It is often laborious to record and analyze the impact information. Therefore, with the use of impact point recognition, the system can help athletes record their training data during training, including ball trajectory, ball drop point, and drop point analysis. This data can help athletes understand their training situation, make targeted technical improvements, and objectively help athletes improve their competitive level.

In traditional spot recognition systems, a large number of sensors, such as vibration sensors, sound sensors, and pressure sensors, are often used. This method requires a lot of hardware and is cumbersome and complicated to implement, so it is often difficult to apply in an extensive range. In recent years, machine vision and image processing technologies have thrived. In particular, target detection and tracking technologies have become more mature. This has enabled the development of spot recognition technology to receive more support. Not only has the accuracy of system recognition increased, but also it is costly. The cost of hardware equipment continues to drop. In the future, the combination of image technology and spot recognition technology will be closer.

This paper proposes a novel algorithm for spot recognition and scoring in table tennis based on dual-channel target motion detection based on the above observations. The algorithm consists of multiple input channels to jointly learn different characteristics of table tennis images. The original image is used as the input of the first channel. Then the Sobel operator is used to extract the first-order derivative feature of the original image, and it is used as the input of the second channel. The table tennis feature information from the two channels is fused and sent to the 3DCNN module. After a fully connected layer, it is finally used to identify the table tennis ball's drop point, compare it with the label's drop point, calculate the error distance, and give a score.

The following are the main contributions of this paper:

1. Aiming at the problem of the ball's falling point, we propose a novel algorithm for identifying and scoring the falling point in table tennis based on dual-channel target motion detection. The input channel is composed of different characteristics of table tennis images.
2. We also use the Sobel operator to extract the first derivative features of the table tennis image, which effectively detect the table tennis's edge in a complex environment.
3. We perform image preprocessing on the video sequence transmitted from the specific table tennis training scene, use Gaussian filtering suppresses image noise, and then convert the color image into a gray image and later into a binary image.
4. We also constructed a data set and conducted experiments. The experimental results show that the method in this paper is superior to some current advanced methods.

## 2. Related Work

In this section, we discuss the literature review in detail under various subsections.

### 2.1. Spot Recognition

The landing point recognition system is an essential branch of the Hawkeye system. When a Ping-Pong game is in progress, the ball's landing information often determines the game's outcome. The Ping-Pong landing point's recognition includes three hardware equipment parts: high-speed cameras, computers, and screen. Among them, the high-speed camera is responsible for collecting multiangle flight data during the sphere's movement, including the speed, angle, rotation, and position. The computer is responsible for establishing a spatial coordinate system with the playing field as the reference system and performing complex data operations to generate three-dimensional images. The screen is responsible for restoring the sphere's trajectory and imaging the falling point in time. The spot recognition system is collaborative development in multiple fields such as machine vision, image processing, and 3D reconstruction. It mainly includes two aspects of technology: one is machine vision technology, which uses multiple cameras to capture images from different perspectives of the ball during movement and realizes the detection and tracking [15–17] of the sphere in the video sequence to obtain the ball's position data. The second is to use computer graphics technology to use the captured position information to restore and analyze the ball's flight state, reconstruct the trajectory, identify the landing point, and display it to the large screen audience.

The spot recognition algorithm's core technical difficulty lies in the accurate detection and positioning of the image's spherical target. It includes various steps: First, the table tennis needs to be detected in the image. Due to table tennis's small size, fast speed, and complex competition environment, tennis balls tend to have minor shape changes. Therefore, it is not easy to obtain good results using the gray image's color and shape features to detect the sphere. In practical applications, it is necessary to combine sports characteristics and comprehensively analyze the number of sports spheres. The second step is to calibrate the camera used in the system. In the spot recognition system, the court is used as a reference to establish a coordinate system to find the relative motion relationship between the sphere and the reference and calculate the sphere based on the camera's calibration parameters (the coordinate data). The third step is the reconstruction of the sphere trajectory. The monocular camera usually does not contain the depth information of the sphere. If you want to fit the three-dimensional trajectory, you need at least binocular vision data. There are mature algorithms for point reconstruction, such as least squares, multiplication, optimization criterion, and methods based on algebraic geometry.

### 2.2. Moving Target Detection

Moving target detection [18, 19] is to detect moving parts (e.g., pedestrians, vehicles, balls, etc.) from the surrounding static environment in the video and extract the detection area frame to determine the moving coordinates target. It is usually divided into two situations: One is that the observer is in a static state. At this time, it is necessary to distinguish the static background area and the moving target area. The research method generally analyzes the moving target's position change in the video sequence before and after the frame. The static area examines the prior knowledge of itself; the second is that the observer is also in a mobile state. At this time, it is necessary to analyze the movement changes of the moving target itself and explore the relative motion relationship between the moving target and the observer in combination with the actual environment for establishment. Traditional moving target detection algorithms include background subtraction, interframe difference, and optical flow. Good results have been achieved in their respective suitable scenarios, but they also have shortcomings. With the development of computer vision theory and computer computing performance improvement, many scholars have improved the above algorithms in combination with actual scenarios. For example, the three-frame difference algorithm based on edge features has solved incomplete holes in the target area. The introduction of optical flow information into the interframe difference method improves detection accuracy and increases computational complexity.

After 2012, convolutional neural networks [20] (CNN) have developed rapidly. In moving target detection scenarios, CNN provides a novel approach, treating sequences in a series of video streams as independent frames. Since 2014, excellent target detection models such as R-CNN (Region-CNN) [21], FastR-CNN [22], and FasterR-CNN [23] have appeared one after another. These methods are based on the idea of classifying and predicting candidate regions. This idea is to improve the detection accuracy of a single frame image. However, because this method needs to generate many candidate regions when processing each frame image and complex calculations are required for each region, the video will yield 30–60 regions per second. This method is slow in actual application and cannot meet the real-time requirements. In response to the real-time application of the problem, the researchers used the idea of regression to propose some efficient and fast detection models, such as YOLO (You Only Look Once) [24] and SSD (Single Shot MultiBox Detector). The YOLO algorithm only needs one CNN operation, provides end-to-end prediction, and improves the detection speed. The video detection frame rate can reach 45FPS, but the detection effect can only be maintained at 63.4% mAP. Because the algorithm is susceptible to the object's scale, the algorithm's generalization ability will become worse when the object's scale changes considerably. The detection accuracy is very low, especially when facing small objects like table tennis.  Figure 1 depicts the principle workflow of this mechanism. The SSD algorithm can extract multiscale features of the image. The algorithm will select the appropriate feature map according to the detected target scale, using extensive features for small targets and minor features for large targets. This way, it dramatically enhances the generalization ability of the algorithm and improves the accuracy of detection.

## 3. Methodology

To accurately identify the table tennis ball's location information, it is necessary to extract and analyze the table tennis ball's complete trajectory and state. First, it is essential to record the table tennis ball's coordinates during the movement and obtain the trajectory coordinates. The most effective way is to perform real-time detection and tracking of the Ping-Pong ball in the video sequence, mark the Ping-Pong ball's position in each frame of the image, and output the position coordinates. Considering that the system in this paper is applied in the particular scene of table tennis training, it is necessary to do image preprocessing for complex application scenes to improve the detecting accuracy and tracking table tennis in the video.

### 3.1. Image Preprocessing

The camera's original video image is generally noisy, which will interfere with the subsequent processing, so it needs to be smoothed to reduce the computational complexity and improve the system's real-time performance. The RGB image transmitted by the camera needs to be digitally converted. To express the image itself with less feature data, interference pixels and void areas usually appear for the detected target area, which needs to be processed by morphological operations. These operations are introduced separately below.

#### 3.1.1. Image Smoothing

To reduce the image noise, it is necessary to smooth the original video data, which is generally achieved by image filtering, preserving the image's detailed features to the greatest extent and filtering out as much mixed noise as possible. Filtering methods for image noise are divided into two categories: linear filtering and nonlinear filtering. There are three commonly used filters: mean filter, median filter, and Gaussian filter. The mean filter is linear. It first calculates the average value of all pixels in the set window area, uses this average value as the anchor point value, and sets all pixels' value in the window as the anchor point value. This method is simple in principle and easy to implement, but it will cause the image to lose much edge information and detailed features. The median filter is nonlinear. First, it calculates the median value of the convolution kernel of all pixels in the set area and then uses this median value as the anchor point value and set the value of all pixels in the window anchor value. This method can effectively save the image's edge information and is very suitable for filtering impulse noise and salt-and-pepper noise.

The Gaussian filter is linear. First, a Gaussian model is calculated based on the Gaussian function's distribution, and then this model is used to achieve convolution and summation of the image. This method has three advantages: one is that the Gaussian function has rotational symmetry and does not change the edge direction of the original image; the second is that the anchor point value is less affected by the distant pixels; the third is to avoid pollution of high-frequency signals. Due to the superior performance of the Guassian filter over the filters, we opted to use it in our proposed work for image smoothing. The Gaussian function is as follows:

(1) $$\begin{array}{c} G\left(x,y\right)=\frac{1}{2\pi \sigma^{2}}{\;e}^{-\left(x^{2}+y^{2}|/|2\sigma^{2}\right)}. \end{array}$$

#### 3.1.2. Digital Image Conversion

There are generally three methods for converting color images into grayscale images: maximum value method, average value method, and weighted average method. In the maximum value method, take the largest pixel value among the three channels of the RGB image as the gray value of the grayscale image:

(2) $$\begin{array}{c} \text{Gray}\left(i,j\right)=\max\left\{R\left(i,j\right),G\left(i,j\right),B\left(i,j\right)\right\}, \end{array}$$

where (*i*, *j*) represents the pixel coordinates, *R*(*i*, *j*) represents the value of the red channel, *G*(*i*, *j*) represents the value of the green channel, *B*(*i*, *j*) represents the value of the blue channel, and Gray(*i*, *j*) represents the gray value.

In the average value method, take the average of the three channels' pixels in the RGB image as the gray image's gray value.

(3) $$\begin{array}{c} \text{Gray}\left(i,j\right)=\frac{R\left(i,j\right)+G\left(i,j\right)+B\left(i,j\right)}{3}. \end{array}$$

In the weighted average method, considering that the human eye has different perceptions of the three primary colors, the pixel values of the three channels are weighted first, and then the average value is taken.

(4) $$\begin{array}{c} \text{Gray}\left(i,j\right)=0.299*R\left(i,j\right)+0.578*G\left(i,j\right)+0.114*B\left(i,j\right). \end{array}$$

Image binarization is to convert a color image or grayscale image to a black and white image, that is, to set the values of all pixels in the image to 0 or 255. This is done to facilitate the subsequent extraction of the target foreground area. First, set the pixel threshold *T*, and set the pixel value of the pixel with the gray value greater than or equal to 255; otherwise, set it to 0.

(5) $$\begin{array}{c} b\left(x,y\right)=\left\{\begin{array}{cc} 255, & g\left(x,y\right)\geq T,\\ 0, & g\left(x,y\right)<T, \end{array}\right) \end{array}$$

where *g*(*x*, *y*) is the input grayscale image and *b*(*x*, *y*) is the output binary image.

#### 3.1.3. Morphological Processing

Morphological processing uses a specific shape of convolution kernel to extract the corresponding shape in the image. Corrosion (as shown in Figure 2) can eliminate boundary points, shrink the image boundary, and then reduce the target area's scope. It is generally used to eradicate meaningless small objects. The formula is as follows:

(6) $$\begin{array}{c} A\Theta B=\left\{x,y|{\left(B\right)}_{xy}\subseteq A\right\}, \end{array}$$

where B represents the convolution kernel, A represents the original image, and the origin is defined in B. The movement process of B and A is similar to the convolution kernel. When the origin of B moves to the pixel (x, y) of image A and the position of B is completely contained in the overlapping area of image A, the pixel point (x, y) of the corresponding output image is allocated as 1; otherwise, the value is 0.

### 3.2. Corner Detection of Tennis Table

The corner point refers to the intersection point produced by the intersection of two edges in the image. In the corner point's local neighborhood, some boundaries belong to two different areas and extend in different directions, as shown in Figure 3. When performing corner detection, it is generally necessary to convert the corner points into points with certain specific characteristics and determine the corner coordinates by detecting the characteristics. The selection of features is usually divided into mathematical features, gray image features, Gradient change characteristics of the image.

The red dots in Figure 4 are the detected corner coordinates.

### 3.3. Sobel Edge Detection Operator

Sobel operator, sometimes called Sobel filter, is used for edge detection in image processing and computer vision images. The Sobel operator is mainly used for edge detection. Technically, it is a discrete differential operator used to calculate the gradient's approximate value of the image brightness function. Using this operator at any point of the image will generate the corresponding gradient vector or its normal vector.

Assuming that the original image is I, the derivation is obtained in the horizontal and vertical directions, respectively.

In the horizontal direction, multiply image I with a matrix whose convolution kernel is an odd number. Generally, the size of the convolution kernel is set to 3. The calculation equation is as follows:

(7) $$\begin{array}{c} G_{x}=\left[\begin{array}{ccc} -1 & 0 & 1\\ -2 & 0 & 2\\ -1 & 0 & 1 \end{array}\right]\times I. \end{array}$$

In the vertical direction, multiply image I with a matrix whose convolution kernel is an odd number. Similarly, the size of the convolution kernel is consistent with the horizontal direction. The calculation equation is as follows:

(8) $$\begin{array}{c} G_{y}=\left[\begin{array}{ccc} -1 & -1 & -1\\ 0 & 0 & 0\\ 1 & 2 & 1 \end{array}\right]\times I. \end{array}$$

Next, square *G*_*x*_ in the horizontal direction and *G*_*y*_ in the vertical direction to get the approximate gradient *G*. The calculation equation is as follows:

(9) $$\begin{array}{c} G=\sqrt{G_{x}^{2}+G_{y}^{2}}. \end{array}$$

### 3.4. Two-Channel Three-Dimensional Convolutional Neural Network

As shown in Figure 5, the dual-channel target motion detection algorithm consists of multiple input channels that jointly learn different features of table tennis images. The original image is used as the input of the first channel. Then the Sobel operator is used to extract the first-order derivative feature of the original image, and it is used as the input of the second channel. The table tennis feature information from the two channels is fused and sent to the 3DCNN module and then to a fully connected layer and is finally used to identify the table tennis ball's drop point. Then we compare it with the label's drop point, calculate the error distance, and give an output score.

As shown in Figure 6, we give the principle of calculating the score of the landing point. Specifically, we use the Euclidean distance to calculate the deviation distance for the predicted landing point and the actual landing point. Since the table is flat, the score calculation can be expressed as follows:

(10) $$\begin{array}{c} \text{Score}=\sqrt{x^{2}+y^{2}}. \end{array}$$

## 4. Experimental Verification and System Implementation

### 4.1. Experimental Environment

Since we use a deep neural network in our model, the computation scale is large and the structure is quite complex. We use Python version 3.6 and Keras 2.1.5 and PyCharm as the IDE to implement the entire model. We conduct an extensive set of experiments on a desktop PC with an Intel Core i7-8700 processor and an NVIDIA GeForce GTX 1080ti GPU. We use an L2 regularizer to regularize the entire network. To speed up the proposed model's performance, we adopt to use the dropout mechanism [25, 26], which randomly drops some neuron and increases the speed of the model along with higher accuracy. The dropout value ranges within {5%, 10%, and 20%}, and we achieved the best result with 20%. We used the Adam optimizer with the learning rate set to {0.01, 0.05, 0.001, and 0.005}. However, we achieved optimal performance when the learning rate was set to 0.001.

The table tennis table uses a standard game table: 76 cm high, 2.74 meters long, and 1.525 meters wide. We use the Hikvision model DS-2DC75201W high-definition high-speed camera; the video frame rate is set to 60 fps with the resolution being 1920 ∗ 1080, and the horizontal viewing angle is set to 60. The camera is installed on the straight line where the table tennis net is located, 1 meter from the lower edge of the table and 1.5 m above the table's surface. On the position above the table's side, we further adjust the camera's shooting angle and focal length to ensure that the ball can be captured and the complete area of the table's right desktop.

### 4.2. Datasets Preprocessing

In this paper, we have collected 100 pieces of game data from table tennis competitions and preprocessed them. Besides, we also obtained 10,000 training images of table tennis placement images. Since this data set comes from real-world competitive competitions, these images are challenging to draw decisions from.

### 4.3. Server System Design

After the system is started, the server first opens the TCP connection and enters the command monitoring state. After the client's connection is established, we start the “heartbeat” detection program to detect whether the client is disconnected abnormally.

If an abnormal disconnect flag occurs, the server ends the connection and tries to connect. Then, return to the monitoring state, analyze the client's JSON file, and get the training server's serving frequency and the number of training rounds. Next, the system obtains the playing video through the RTSP protocol. Also, the model executes the image preprocessing program, including image filtering, image feature conversion, corner detection of the table tennis table, and selection of the region of interest. The proposed approach then detects and tracks the sports table tennis in the region of interest, records and saves the ball's centroid coordinates, and uses the ball track coordinates of a whole round to track the trajectory. The equation is fitted and reconstructed, the coordinates of the table tennis's drop point are analyzed, the area classification of the drop point is obtained, the result is returned to the client, and the monitoring state is reentered until the program execution ends.

### 4.4. Experimental Results

Tables 1 and 2 illustrate the gratifying results of the proposed model.

From the perspective of table tennis, the algorithm in this paper achieves the best results at 0 degrees, 36 degrees, and 126 degrees. Also, we find that the performance of table tennis recognition is the worst at 90 degrees. Nevertheless, this paper's algorithm still achieved an average recognition accuracy rate of 77.42, achieving satisfactory performance. This article also discusses the impact of different numbers of training samples on the experimental results. We divided the data set into 7 different proportions. When 1% of training samples are used, the table tennis placement score of the algorithm in this paper is 15.32. When increasing the training samples until it reaches 20%, the drop point score drops sharply, proving that the algorithm's performance is greatly enhanced with the increase of training samples.

### 4.5. Ablation Experiment

In this section, we discuss the influence of dual channels on the experimental results. In this paper, the dual channels are divided into three groups of experiments. The first group is the single channel of the original image. The second is the single channel of the Sobel operator. The third is the double-channel algorithm proposed in this paper.

It can be seen from Table 3 that the performance of using the Sobel operator is significantly better than that of using the original image. Also, the dual-channel algorithm proposed in this paper is far more superior to the two single-channel algorithms, which proves the effectiveness and the excellent performance of the proposed model.

## 5. Conclusion

This paper proposes a novel algorithm for spot recognition and table tennis scoring based on dual-channel target motion detection. The algorithm consists of multiple input channels to jointly learn different characteristics of table tennis images. The original image is used as the input of the first channel. Then the Sobel operator is used to extract the first-order derivative feature of the original image, and it is used as the input of the second channel. The table tennis feature information from the two channels is fused and sent to the 3DCNN module. The output is then fed into a fully connected layer. It is finally used to identify the table tennis ball's drop point, which further compares it with the drop point of the label, calculates the error distance, and finally generates an output score. This article mainly realizes the functions of table tennis's spot recognition and regional scoring. It has high recognition accuracy and real-time performance and can provide scientific auxiliary suggestions for sports teams.

## Figures and Tables

**Figure 1:** YOLO (You Only Look Once) architecture.

**Figure 2:** Image corrosion operation process.

**Figure 3:** Different types of corner points.

**Figure 4:** Table corner detection results.

**Figure 5:** Two-channel three-dimensional convolutional neural network.

**Figure 6:** Score calculation diagram.

**Table 1:** Scoring result of falling-point prediction in table tennis (less is better).

Training samples (%)	Score (less is better)
1	15.32
5	14.96
10	13.21
20	10.11
30	8.25
50	4.5
100	**2.21**

**Table 2:** The recognition rate of table tennis.

Angle (°)	Recognition rate
0	92.3
36	85.2
54	72.3
72	71.3
90	56.6
126	86.8

Average recognition rate	77.42

**Table 3:** Ablation experiment (higher is better).

Training samples	Average recognition rate
Original	61.85
Sobel	65.98
Dual-channel	**77.42**

## Data Availability

The data used to support the findings of this study are included within the article.
